# Diffuse and multifocal nephrogenic adenoma with Familial Mediterranean Fever: a case report with molecular study

**DOI:** 10.1186/s13000-015-0344-7

**Published:** 2015-07-16

**Authors:** Noriyoshi Ishikawa, Chika Amano, Takeshi Taketani, Koji Kumori, Yuji Harada, Hisayuki Hiraiwa, Kayoko Itamura, Riruke Maruyama

**Affiliations:** Department of Pathology (Organ Pathology Unit), 89-1 Enya, Izumo, Shimane 693-8501 Japan; Department of Pathology (Functional Pathology Unit), Shimane University School of Medicine, Shimane, 693-8501 Japan; Department of Pediatrics, Shimane University School of Medicine, Shimane, 693-8501 Japan; Department of Digestive and General Surgery, Shimane University School of Medicine, Shimane, 693-8501 Japan; Laboratory of Surgical Pathology, Shimane University Hospital, Shimane, 693-8501 Japan; Department of Pediatrics, Eastern Shimane Rehabilitation Hospital, Shimane, 693-8501 Japan

**Keywords:** Urinary tract, Nephrogenic adenoma, Familial Mediterranean fever, MEFV gene mutation

## Abstract

Nephrogenic adenoma, also referred to nephrogenic metaplasia, is a benign proliferative lesion of urothelium, usually associated with chronic physical stimuli or inflammation. Familial Mediterranean fever is an inherited autosomal recessive disease characterized by recurrent short episodes of fever. The site of mutation is found in *MEFV* gene which controls inflammatory responses. We have experienced a case of nephrogenic adenoma in a 16-year-old girl with Familial Mediterranean Fever, showing proliferative lesions diffusely in the urinary bladder and multifocally in the other parts of urinary tract. These lesions disappeared after colchicine treatment. We searched for *MEFV* gene mutation using the specimen from the resected urinary bladder and detected heterozygous mutation of E148Q. There is a possibility that control of inflammation caused by the surgery for vesicoureteral reflux in the local site didn’t work well on the background of heterozygous mutation of *MEFV* gene, and as a result, nephrogenic adenoma appeared. This is the first report of a combination of two rare diseases. We have to be aware that nephrogenic adenoma can occur in association with Familial Mediterranean Fever, and the former condition should be taken into consideration when rendering a correct pathological diagnosis.

## Background

Nephrogenic adenoma is a benign tumor-like lesion of the urinary tract, characterized by a papillary and tubular proliferation of cuboidal cells similar to the epithelial cells of distal renal tubules. It occurs anywhere in the urinary tract, but it is most frequently found in the bladder [1]. It was first described in 1949 by Davis [2], and originally thought to arise from a remnant of mesonephric tissue or metaplasia of the urothelium in response to chronic irritation and mucosal damage. Currently, it is known that exfoliated and implanted renal tubular cells into the urinary tract mucosa form the disease [3]. The most common histological pattern is a proliferation of small tubules composed of a single layer of cuboidal epithelium. These tubules are often surrounded by a hyalinized basement membrane and contain blue mucin in the lumens. It may also grow in papillary, cystic or solid pattern. Hobnail cells may be seen in papillary growth areas. In cystic pattern, colloid-like eosinophilic secretion or blue-tinged mucin is frequently observed [1]. Occasionally, clear cells or signet-ring cells can be seen in solid area, which could be confused with poorly differentiated adenocarcinoma. Although it arises commonly in adults, approximately 10 % of the patients are children, and several cases of even younger patients have been reported in the literature [4–7].

Familial Mediterranean fever (FMF) was first reported as ‘benign paroxysmal peritonitis’ in 1945 [8] and the current name of the disease was proposed in 1958 [9]. Most of the reported cases are autosomal recessive disease characterized by recurrent short episodes of fever and pain due to serosal inflammation [10]. In 1997, a responsible gene was cloned and named *MEFV*. It encodes a protein pyrin that controls inflammation [11, 12]. Frequent mutations have been found in M694V, M694I, V726A, M680I of exon10 and, E148Q of exon 2 [13]. This disease is most common in the periodic fever syndrome and characterized by high effectiveness of colchicine administration [14]. We present the first rare case of nephrogenic adenoma secondary to FMF, occurring throughout the urinary tract. There has been no such a report in the literature and also, it is very rare that nephrogenic adenoma involves almost the whole mucosa of urinary tract.

## Case presentation

A 16-year-old girl presented with disturbed consciousness and was admitted to our hospital under the diagnosis of hypertonic dehydration. During the pregnancy (32 weeks of gestational age) of her mother (29-year-old at that time), she was born by an urgent cesarean section for a shock state due to rupture of the right ovary metastasized by gastric cancer. The mother died of gastric cancer at the age of 33. The patient presented with fetal distress syndrome at birth, and thereby had sequelae such as developmental and mental retardation and epilepsy. Thereafter, she repeated urinary tract infection (UTI) caused by vesicoureteral reflux. However, even after the surgery, remittent fever came to arise twice or three times a month, but causative bacteria could not be identified by either urinalysis or urine culture. Leukocytosis and slightly high level of CRP (C-reactive protein) continued to be observed. Immunological test revealed slightly low value of CH50. On admission, swelling of left kidney was pointed out with the abdominal computed tomography. Abdominal ultrasonography revealed the left hydroureteronephrosis associated with a bladder mass. In the meantime, the tumor gradually enlarged to fill the whole lumen of the bladder, and she finally developed bilateral hydroureteronephrosis. As a result, the patient underwent total cystectomy followed by cutaneous ureterostomy.

Grossly, papillary or villous mass totally occupied the bladder lumen measured 7 cm in the maximum diameter (Fig. 1). Histologically, various patterns of structure were observed. The most predominant pattern was villous architecture with delicate core vessels, composed of hobnail tumor cells with high N/C ratio (Fig. 2a and b). Areas of small gland proliferation and cystic change were also seen, both of which had colloid-like eosinophilic secretion in the lumens (Fig. 2c and d). In addition, proliferation of microtubules was also observed, simulating　poorly differentiated adenocarcinoma or signet-ring cell carcinoma (Fig. 2e and f). Mucin was identified in PAS/Alcian-blue double staining (Fig. 2g).

**Fig. 1:** Gross appearance of resected bladder; Papillary or villous projections are observed in the lumen of the bladder (**a**: whole image, **b**: cut surface)

**Fig. 2:** Histologic appearances of nephrogenic adenoma. **a** The tumor proliferated in very thin villous pattern with delicate core vessels. **b** Hobnail structure of the tumor cells with high N/C ratio was identified. Various size of glands were seen. **c** Comparatively small glands and (**d**) large glands with cystic change. Both of them had colloid-like eosinophilic secretion in the lumens. **e**, **f** Microtubular structures were also observed. They were quite similar to poorly differentiated adenocarcinoma or signet-ring cell carcinoma in part. **g** Mucin could be identified with PAS/Alcian-blue double stain. **h** Vimentin was diffusely positive with immunohistochemical analysis. **i**, **j** PAX8 was diffusely positive in all histological structures of nephrogenic adenoma. **k** PAX2 was also positive. **l** Ki-67 postive cells were very few

Formaline-fixed, paraffin-embedded (FFPE) tissue was cut into sections of 3 μm thickness and immunostain was performed with the primary antibodies (Table 1) according to the manufacturers’ instructions and visualized employing Ventana BenchMark ULTRA immunostainer (Ventana Medical Systems, USA). Immunohistochemically, the tumor cells were positive for CK7, α-methyl-acyl-CoA racemase (AMACR), CA19-9, vimentin (Fig. 2h), PAX8 (Fig. 2i and j), PAX2 (Fig. 2k), CD138 and CD10, and negative for p63 and prostate specific protein (PSA). The Ki-67-positive cells were very few (Fig. 2l). In the background, cystitis glandularis with hypeplastic urothelium was observed with variety of inflammatory cell infiltration, including neutrophils, mast cells and plasma cells. These histological findings were consistent with nephrogenic adenoma. After surgery, papillary lesion recurred in the bilateral renal pelvises and nearby ureters, but most of the recurrent lesions disappeared by colchicine treatment.

**Table 1:** Summary of antibodies employed in this case

Marker	Antibody	Source	Dilution
CK7	Anti-Human Cytokeratin 7, monoclonal, Clone OV-TL 12/30	Dako, Glostrup, Denmark	1:100
AMACR	Anti-Human P504S, rabbit monoclonal, Clone 13H4	Dako, Glostrup, Denmark	1:100
CA19-9	Anti-CA19-9, mouse monoclonal, Clone BC/121SLE	Biocare, Concord, USA	1:100
Vimentin	Anti-Vimentin, mouse monoclonal, Clone V9	Dako, Glostrup, Denmark	1:100
CD138	Anti-Human CD138, monoclonal, Clone MI15	Dako, Glostrup, Denmark	1:50
CD10	Anti-CD10, rabbit monoclonal, Clone SP67	Roche, Basel, Switzerland	1:1 (prediluted)
p63	Anti-p63, mouse monoclonal, Clone BC4A4	Biocare, Concord, USA	1:200
PSA	Anti-Human Prostate-Specfic Antigen, Clone ER-PR8	Dako, Glostrup, Denmark	1:50
PAX8	Anti-Pax8, mouse monoclonal, Clone BCl2	Biocare, Concord, USA	1:1 (prediluted)
PAX2	Anti-Pax2, rabbit monoclonal, Clone EP3251	Abcam, Cambridge, UK	1:1000
Ki-67	Anti-Ki67, rabbit monoclonal, Clone 30-9	Roche, Basel, Switzerland	1:1 (prediluted)

Considering the effectiveness of colchicine treatment, we searched for MEFV gene mutations. In Japan, about 100 cases of FMF have been reported with frequent mutations found in E148Q (exon2) and M694I (exon10), so we searched for these mutations using formalin fixed samples of this case. Genomic DNA was extracted from 10 FFPE sections of 10 μm thickness using QIAamp DNA FFPE tissue kit (QIAGEN, Venio, Netherland) according to the manufacturer’s recommendations. The following PCR primers were used for amplification of *MEFV* (exon2 and, exon10).

5’-AGATGATTCCGCAGCGTCCA-3’(exon2-F),

5’-AGGCTTGCCCTGCGCGTCCA-5’(exon2-R),

5’-TCCTGGGAGCCTGCAAGACA-3’(exon10-F),

5’-AAAGAGCAGCTGGCGAATGT-3’ (exon 10-R).

Thermal cycling conditions were 5 min at 94 °C, followed by 35 cycles of 94 °C for 30 s, 62 °C(exon 2) or 56 °C (exon 10) for 30 s and 72 °C for 1 min followed by a final incubation at 72 °C for 7 min. The PCR products were purified using QIAquick PCR purification kit (QIAGEN, Venio, Netherland). After purification of PCR products, analyses by capillary electrophoresis on a 3130 Genetic Analyzer (Applied Biosystems, Foster City, CA) were performed. Sequence electropherograms were analyzed by Sequence Analysis 5.2 software (Applied Biosystems). As a result, we could not find any mutations in exon 10 but a heterozygous mutation of E148Q was detected in exon2 (Fig. 3).

**Fig. 3:** Sequence analysis of exon 2. **a** Heterozygous point mutation of E148Q was detected. **b** Enlarged view of mutation area. Spine of blue line is C: cytosine and those of black line are G: guanine of base DNA

## Discussion

In the past, nephrogenic adenoma was thought to arise from the remnant of embryogenic mesonephric tissue in the urinary tract, or from metaplastic change of urothelium due to inflammation or injury. In 1981, Bhagavan et al. examined nephrogenic adenoma morphologically with electron microscopy and found the presence of Tamm-Horsfall protein [15]. They revealed that this lesion was of mesonephric origin rather than of metanephric. Based on the fact that the nephrogenic adenoma often occurs in patients who received kidney transplantation, Mazal et al. in 2002 [3] made a research into the origin of nephrogenic adenoma. They analyzed X and Y chromosomes employing fluorescence in situ hybridization. In the cases of male recipients from female donors, the cells of nephrogenic adenoma had XX chromosome pattern, On the contrary, in the cases of female recipients from male donors, the cells had XY chromosome pattern. These results indicated that origin of nephrogenic adenoma was donor-derived renal cells [3]. Moreover they thought nephrogenic adenoma in extrarenal organs like urinary bladder was caused by proliferation of cells of renal origin, and showed positive immunostaining of PAX2 [16]. PAX2 is a transcriptional factor in development and expressed in renal tubular cells and parietal cells of the Bowman’s capsule of gromerulus [16]. PAX2 has recently been considered to be one of the useful markers for nephrogenic adenoma [16]. “　PAX8, another transcriptional factor, expressed in renal cells is also positive in nephrogenic adenoma [17]. It is currently thought that dislodged renal tubular epithelial cells are transplanted into the urinary tract mucosa and engraftment occurs, resulting in the disease [3]. In the present case, repeated urinary tract infection might have contributed to the development of nephrogenic adenoma. We consider that occurrence of the tumor in renal pelvis of both sides after bladder extraction supported this hypothesis.

About 10 % of the cases with nephrogenic adenoma occur in pediatric age [1], and show the same morphological and immunohistochemical features as adult cases [18]. They occur under the specific pathological conditions such as Turner's syndrome [4] or prune belly syndrome [5]. Multifocal [6] and/or diffuse [7] lesions have also been reported. FMF is known to cause inflammatory conditions such as peritonitis, pleurisy, arthritis, erysipelas-like erythema and pericarditis. Responsible gene of FMF located at chromosome 16p13.3 encodes a pyrin/marenostrin protein composed of 781 amino acids and consists of 10 exons [11, 12]. Usually, pyrin has N-terminal PYRIN domain and C-terminal B30.2 domain. Activity of caspase-1 is regulated by ASC (apotosis-associated speck-like protein which contains a caspase recruitment domain) which bound to PYRIN domain and, B30.2 domain also regulates activity of IL-1β by directely inhibition of caspase-1 activation [19, 20]. Major mutations of FMF are found in E148Q in exon 2, and M894V, M694I, V726A, and M680I in exon 10 of *PYD* [21, 22]. If there is a mutation in exon 10, the diagnosis of FMF can be confirmed. Additionally, if mutations in the other exons, including heterozygous mutation are detected, colchicine can be utilized not only for a treatment, but also for a diagnosis of FMF variant [23]. In FMF variants, mutations in exon 1 (E84K), exon 2 (L110P, E148Q, R202Q, G304R), exon 3 (P369S, R408Q) and exon5 (S503C) are known. It is believed that inflammation is provoked by missense mutations of *PYRIN* gene which result in loss of suppressive function of inflammasome and increase of IL-1β production [19, 20]. In our case, only one heterozygous mutation of E148Q (exon2) was observed. There is a report that this mutation was seen in 20 % of Japanese patients [24], but the present case was diagnosable as FMF variant, because treatment with colchicine was very effective. We did not search for other mutations on the chromosome, because most of them are limited at E148Q (exon2) and, M694I (exon 10) in the Japanese patients. Pyrin, located in microtubules and actin [25], is a protein highly expressed in white blood cells. They are coded by MEFV gene which regulates inflammatory response by interacting with the cytoskeletons and mutation of this gene probably decreased or deleted its function [25]. Colchicine also has a function to inhibit the polymerization of microtubules (tubulin). In the present case, not only white blood cells but also the tumor cells of nephrogenic adenoma were positive for vimentin. This suggests the possibility of expression of tubulin (component of cytokelaton). Many of the FMF cases are autosomal recessive, and the symptoms are less likely to occur in heterozygous mutation of E148Q (exon 2), so that the patient might have different mutations to cause the symptoms.

## Conclusion

To our knowledge, this is the first report of nephrogenic adenoma in a FMF patient. We speculate that control of inflammation in the local site didn’t work well on the background of heterozygous mutation of *MEFV* gene, thus, being triggered by mechanical operation of urinary tract, proliferation of nephrogenic adenoma was induced. However, an accumulation of the similar cases is mandatory to clearly elucidate the mechanisms of the disease. Furthermore, we should be aware that nephrogenic adenoma can occur in FMF patients to render a correct diagnosis.

## Consent

Written informed consent was obtained from the patient’s father for publication of this Case report and any accompanying images. A copy of the written consent is available for review by the Editor-in-Chief of this journal.
